# History of Prostatitis Is an Independent Risk Factor for Erectile Dysfunction: A Cross-Sectional Study

**DOI:** 10.1155/2020/8964673

**Published:** 2020-10-17

**Authors:** Chengquan Ma, Zhonglin Cai, Jian Xiong, Hongjun Li

**Affiliations:** Department of Urology, Peking Union Medical College Hospital, Peking Union Medical College, Chinese Academy of Medical Sciences, Beijing 100730, China

## Abstract

**Purpose:**

To determine the role of history of prostatitis (HP) as an independent risk factor for erectile dysfunction (ED) in Chinese adult males.

**Methods:**

We conducted an online survey using a crowd-sourced questionnaire in Chinese adult males. The participants were separated into two groups as adult participants with HP and with no history of prostatitis (NHP) according to the medical history record. As diagnosis criteria of ED, we used the 5 questions of the International Index for Erectile Function (IIEF-5). The general data including height, weight, monthly income, academic background, smoking history, alcohol drinking, marital status, conjugal affection, and other disease history was asked and recorded. The relationship between HP and ED using the chi-square test and logistic regression analyses was investigated and analyzed.

**Results:**

In total, 1873 participants answered the questionnaire. 95 participants in the HP group and 1778 participants in the NHP group were included in this study. The rate of participants with HP was 5.343%. ED was found in 68.4% of the HP group and 43% of the NHP group (*p* < 0.001). Regression analysis showed that participants in HP were more likely to have ED (OR 2.135, 95% CI 1.266–3.60) after adjusting for the participant's age, body mass index (BMI), monthly income, academic background, smoking history, alcohol drinking, marital status, conjugal affection, BPH, hypertension, and diabetes mellitus, when compared with NHP.

**Conclusions:**

The present study indicated a high prevalence of ED in Chinese adult males with history of prostatitis, and HP is an independent risk factor for erectile dysfunction.

## 1. Introduction

As a high proportion of diseases in the urology clinic, prostatitis could cause great distress to the healthy life of men in many aspects. Previously, we conducted a study based on questions and answers and the judgment of the urologist on the diagnosis of chronic prostatitis (CP) which is a most common category of prostatitis and found that the occurrence was 25.3% for all life risks of CP in Chinese males aged 40 to 81 years [1]. Prostatitis is clinically complex and the etiologically unclear, making it difficult to diagnose prostatitis with certainty and choose the effective treatment, increasing the difficulty for urology in the clinic practice [2], and its impacts on sexual function (SF) are usually overlooked [3].

Erectile dysfunction (ED) is a common form of dysfunction for men's sexual health, which represents an increasing health concern which impairs the quality of life of men globally. ED is a symptom of a variety of pathologies, including the combined effect of psychological, hormonal, neural, and vascular pathways that can achieve and maintain an erection. Therefore, according to their erectile dysfunction caused by different etiological factors, it usually includes one or more disorders of endocrine, nerve, blood vessel, structure, and psychiatric causes; however, it is difficult for clinicians to distinguish between the two due to their heavy interconnection [4]. It is not clear what the risk factors are to predict ED in patients. Previous research pointed out that risk factors independently related to ED include age, diabetes, hypertension, lower urinary tract symptoms, depression/anxiety, and benign prostate hyperplasia [5–9].

ED and prostatitis have high morbidity and prevalence among men, often becoming apparent over the third decade of life. The coexistence of these conditions is interesting in that evidence suggests a link between prostatitis and ED though the reason is unclear. One study had shown that tadalafil, a classic drug for ED, is also effective for treating prostatitis [10]. In recent years, lots of articles have revealed that a high prevalence of ED ranges from 15.0% to 40.5% among patients with CP/CPPS in China; it is not enough to explain the relationship based on the current research data [11, 12]. Limited studies also found the opposite result that there is no significant relationship between prostatitis and ED [13–15]. Therefore, the relationship between prostatitis and ED remains controversial.

However, all of these studies only enrolled cases with CP/CPPS as the study subject. There is no study to investigate the effect of HP on erectile function for adult men. Therefore, we conducted the present study to examine the prevalence rates of ED in participants with HP and determine the association of ED with HP in China using a crowd-sourced online population-based dataset. After reviewing the literature, we know that this is the first complete study to evaluate the links between HP and ED.

## 2. Methods

### 2.1. Research Plan

We conducted the present cross-sectional study between October 2019 and November 2019. Data from all participants were collected at the online questionnaire in China. All participants with or without prostatitis underwent a clinical evaluation involving a medical history and were also asked to fill out the questionnaire to get the following information: (1) participant's general information, including the age, weight, height, monthly income, academic background, smoking history, alcohol drinking, marital status, conjugal affection, BPH, hypertension, and diabetes mellitus. The monthly income is divided into four levels (¥/month): <2000, 2000~5000, 5000~10000, and >10000; academic background is divided into four levels: ≤junior high school, high school, college, and ≥college; smoking history and alcohol drinking is defined as having smoked or drank in the last six months; marital status is divided into three types: married, single, and divorced or bereaved; and conjugal affection is divided into three types: good, normal, and bad.

(2) We used the first 5 questions of the International Index of Erectile Function 5(IIEF-5) score to assess the erectile function (EF), and ED was diagnosed with score < 22 points [16]. The participants were separated into two groups as cases with a history of prostatitis and with no history of prostatitis. We first introduced the content and plan of the survey to the participants in detail. All participants expressed full understanding of the content and importance of the survey and voluntarily filled out the questionnaire within 20-30 minutes. The data completed by all participants was independently entered and checked by two independent investigators to guarantee the accuracy of the questionnaires. Local ethical approval was obtained from the Ethics Committee of the Peking Union Medical College Hospital. We again explained about the study to participants, who filled out the informed consent form before inclusion in the study. Participants were evaluated according to inclusion and exclusion criteria of the study which are shown below.

### 2.2. Cases' Inclusion Criteria and Exclusion Criteria

The inclusion criteria covered are as follows: (1) according to the diagnostic criteria of the NIH prostatitis classification system, at least one urologist had diagnosed the participants with any type of prostatitis in the hospital to improve the effectiveness of the diagnosis; (2) participants who were diagnosed with prostatitis had recovered from the symptoms more than 6 months; (3) age > 18 years; and (4) have a long-term stable sexual partner.

The exclusion criteria are as follows: (1) diseases that mainly affect SF, including severe mental illness, coronary artery disease that cannot be effectively controlled, severe spinal cord injury, and failure to effectively control endocrine diseases; (2) oral or injection of medicament may influence SF within past 3 months, including phosphodiesterase type-5 inhibitors (sildenafil, tadalafil, or vardenafil), Chinese medicine for changing sexual function, hormone drugs (testosterone undecanoate or estradiol), aromatase inhibitor (tamoxifen or clomiphene), and psychotropic drugs (such as sertraline); (3) a history of pelvic or perineal surgery, congenital malformations of the urogenital system, including testicular tumors, bladder tumors, prostate cancer, and other malignant tumors that may affect sexual function; and (4) currently suffering from prostatitis disease without recovery in symptoms were also excluded.

### 2.3. Statistical Analysis

We applied SPSS 22.0 (IBM Corp., Armonk, NY, United States) to conduct the statistical comparison. We then investigated the relationship between HP and ED using Student's *t*-test or the chi-square test. Logistic regression analysis, with ED as the dependent variable and age, BMI, monthly income, academic background, smoking history, alcohol drinking, marital status, conjugal affection, BPH, hypertension, and diabetes mellitus as independent variables, was used to analyze the associations between these factors and the occurrence of ED in participants with prostatitis.

## 3. Results

### 3.1. Baseline Characteristics of Cases

The distributions of demographic characteristics among HP and NHP groups are shown in Table 1. A total of 95(the rate of participants with HP was 5.343%) cases in the HP group and 1778 participants in the NHP group were included in the research, with a mean age of 33.46 ± 10.84 years and 30.59 ± 9.66 years, respectively. BMI (*p* = 0.094) and monthly income (*p* = 0.709) were found to have no statistical differences between the two groups. The academic background, smoking history, alcohol drinking, marital status, conjugal affection, BPH, hypertension, and diabetes mellitus of cases among HP and NHP were different (all *p* < 0.05).

### 3.2. The Prevalence of ED

The mean scores of IIEF-5 among HP and NHP groups are 17.53 ± 5.94 and 20.71 ± 7.62, respectively (*p* < 0.001). The prevalence of ED among participants with HP was higher than these participants without HP. ED was found at 68.4% of the HP group and 43% of the NHP group (*χ*^2^ = 68.545, *p* < 0.001).

### 3.3. OR between HP and NHP Groups

As compared with the NHP group, regression analysis indicated that risk of ED in the HP group was 2.135 (95%CI = 1.266–3.60, *p* = 0.004) times greater than that in the NHP group after adjusting for the participant's age, BMI, monthly income, academic background, smoking history, alcohol drinking marital status, conjugal affection, BPH, hypertension, and diabetes mellitus (Table 2). We can know that a man with history of prostatitis was more likely to have ED, and it is an independent risk factor for ED.

## 4. Discussion

The links between erectile dysfunction and prostatitis have recently attracted much attention, but the associations of ED with HP remain unclear. In this article, we revealed that OR for HP in participants with ED was 2.135 when compared with that for NHP, after adjusting for participants' age, BMI, monthly income, academic background, smoking history, alcohol drinking marital status, conjugal affection, BPH, hypertension, and diabetes mellitus. The results of the present research showed that compared with no history of prostatitis alone, the history of prostatitis group was significantly associated with ED and HP was an independent risk factor for erectile function. Thus, we can know that erectile function could be affected in a man with HP.

Sexual dysfunction is often associated with prostatitis though limited studies claim that there is still some controversy. Our team had conducted a pooled study which showed that the prevalence of sexual dysfunction for adult males with chronic prostatitis was high up to 62% [17]. ED is one of the most common types of sexual dysfunction; previously, a meta-analysis found that cases with chronic prostatitis have an increased risk of ED compared the control group (pooled OR 3.02, 95% CI: 2.18–4.17) [18]. Subsequently, increasing evidences indicated that there is a relationship between CP and ED. In this study, we selected participants who were diagnosed with any type of prostatitis and found that the prevalence of ED among participants with HP was higher than these participants without HP (68.4% in the HP group and 43% of the NHP group, *p* < 0.001). These results remind physicians to realize that erectile dysfunction for participants with HP could be affected even though they may have recovered. However, the underlying pathophysiological mechanisms are still unclear.

Erectile dysfunction is usually caused by a variety of factors, including inflammation of the prostate and psychological disorders [19]. ED-related risk factors were also found highly prevalent in male with prostatitis [20]. A large number of studies had shown that prostatitis patients are often complicated by psychological disorders due to pain and urination disorders, and these problems may reduce the sexual desire and frequency of sexual intercourse [21–23]. Comprehensive or mixed factors of endocrine, neurogenic, vasculogenic, and psychological factors may play an important role in the pathogenesis of sexual dysfunction caused by prostatitis.

Endothelial dysfunction or arterial stiffness due to prostatitis problems may be related to increased risk factors for ED [20]. Patients with chronic prostatitis were more likely to have vascular endothelial cell damage compared to normal males [20]. During the inflammation of prostatitis, a large number of inflammatory mediators can be released, which may lead to disorders of smooth muscle contraction and relaxation. At the same time, these inflammatory mediators often disrupt the process of microvessel formation and reduce endothelial function. These two factors are likely to prevent effective penile tissue from being filled with blood, thus the decline in the ability to maintain an erection [24]. Neurologic and endocrine factors are also disordered physiological processes associated with ED in patients with prostatitis [25]. Previous studies have indicated that the incidence of nitric oxide-mediated vascular endothelial dysfunction in patients with CP is higher than that in the normal population [20], which may cause ED in patients with HP.

Psychological factors may also be the link to a relationship between prostatitis and sexual function [26]. Furthermore, psychological comorbidities are common in males with prostatitis, and it may be a factor involved in the mechanism of impaired erectile function [27]. In psychological aspects, the most common of these risk factors are anxiety or depression, which can have an adverse effect on sexual function [26, 28]. Patients with prostatitis have a high incidence of sexual dysfunction due to psychological reasons, and patients with prostatitis have more severe stress, depression, anxiety, and adverse impairment of sexual function [29, 30]. These mental illnesses can also cooperate with pain symptoms and urination disorders to jointly disrupt the sexual behavior and erectile function [31]. Thus, we can infer that the role of psychological factors in the pathogenesis of ED is involved in participants with prostatitis for a long time even though they may have recovered.

This study is limited by the cross-sectional design as response to the additional follow-up survey was voluntary. Previously published articles had reported the prevalence of ED at 18% and 37%, in the United States and the Republic of Korea, respectively [8, 32]. Our team also found that prevalence of ED was 40.56% in middle-aged males [33]. In the present study, the mean score of IIEF-5 in NHP groups was 20.71 ± 7.62, and the prevalence of ED among participants in NHP was high up to 43%. The reason for this difference may be as follow: as certain parts of the questionnaire include sensitive questions, some participants might have answered inaccurately; because the sample is based on a highly self-selective online population and completing the questionnaire is very time-consuming, it is easy to cause selection bias to a certain extent; older people use the internet less frequently; participants with low sociocultural status or fear of new technologies may have an impact on the quality of the questionnaire. Another shortcoming due to the limitations of the online questionnaire is that we did not perform subtype analysis for each type of prostatitis. This cross-sectional study did not adequately and effectively evaluate the psychological factors through the psychological questionnaire score, as this is a possible influencing factor and should be included in future studies.

## 5. Conclusion

This article was to assess the effects of HP on erectile function in adult men. We find that men with HP are more likely to develop ED compared to the general population in the future. For urologists, the negative influence on erectile function should get more attention with regard to men with HP. Further study is required to explore the relationship between ED and HP.

## Figures and Tables

**Table 1:** Demographics and clinical characteristics between HP and NHP groups.

Parameters	HP (*n* = 95)	NHP (*n* = 1778)	*p*
Age (years)	33.46 ± 10.84	30.59 ± 9.66	0.005∗
BMI (kg/m^2^)	23.04 ± 3.16	22.44 ± 3.37	0.094∗
Monthly income (¥/month)			0.709^#^ (*χ*^2^ = 1.383)
<2000	12 (6.7%)	168 (93.3%)	
2000~5000	21 (5.1%)	394 (94.9%)	
5000~10000	27 (4.5%)	574 (95.5%)	
>10000	35 (5.2%)	642 (94.8%)	
Academic background			0.014^#^ (*χ*^2^ = 10.648)
≤Junior high school	13 (8.7%)	137 (91.3%)	
High school	20 (7.8%)	235 (92.2%)	
College	51 (4.1%)	1199 (95.9%)	
≥College	11 (5.0%)	207 (95.0%)	
Smoking history			<0.001^#^ (*χ*^2^ = 68.545)
Yes	43 (7.5%)	531 (92.5%)	
No	52 (4.0%)	1247 (96%)	
Alcohol drinking			<0.001^#^ (*χ*^2^ = 43.144)
Yes	58 (10.1%)	518 (89.9%)	
No	37 (2.9%)	1260 (97.1%)	
Marital status			<0.001^#^ (*χ*^2^ = 45.519)
Married	51 (5.2%)	935 (94.8%)	
Single	31 (3.7%)	801 (96.3%)	
Divorced or bereaved	13 (23.6%)	42 (76.4%)	
Conjugal affection			<0.001^#^ (*χ*^2^ = 115.506)
Good	58 (4.5%)	1229 (95.5%)	
Normal	22 (33.3%)	44 (66.7%)	
Bad	15 (2.9%)	505 (97.1%)	
BPH			<0.001^#^ (*χ*^2^ = 68.545)
Yes	18 (26.9%)	49 (73.1%)	
No	77 (4.3%)	1729 (95.7%)	
IIEF-5	17.53 ± 5.94	20.71 ± 7.62	<0.001^∗^
ED			
Yes	65 (68.4%)	764 (43%)	<0.001^#^ (*χ*^2^ = 23.679)
No	30 (31.6%)	1014 (57%)	

HP: history of prostatitis; NHP: no history of prostatitis; BMI: body mass index; BPH: benign prostate hyperplasia; IIEF-5: the first 5 questions of the International Index for Erectile Function; ED: erectile dysfunction. ^∗^*t* − test. ^#^Chi-square test.

**Table 2:** Multivariate logistic regression analysis of the influence of HP and other factors on prevalence of ED in men.

Variable	*β* value	Wald *χ*^2^	OR	95% CI	*p*
Age (years)	0.012	3.602	1.012	1.0-1.024	0.049
BMI (kg/m^2^)	0.132	4.588	1.141	1.011-1.288	0.04
Monthly income (¥/month)	-0.3	22.519	0.741	0.654-0.838	<0.001
Academic background	-0.387	17.912	0.679	0.568-0.813	<0.001
Smoking history	0.362	8.32	1.436	1.123-1.835	0.004
Alcohol drinking	0.289	5.638	1.336	1.052-1.696	0.018
Marital status	-0.137	1.144	1.147	0.892-1.474	0.285
Conjugal affection	0.611	170.293	1.843	1.681-2.02	<0.001
BPH	0.687	4.123	1.988	1.024-3.86	0.042
Hypertension	0.736	9.751	2.087	1.315-3.311	0.002
Diabetes mellitus	1.635	23.566	5.130	2.651-9.927	<0.001
Prostatitis	0.758	8.085	2.135	1.266-3.60	0.004

HP: history of prostatitis; BMI: body mass index; BPH: benign prostate hyperplasia; IIEF-5: the first 5 questions of the International Index for Erectile Function; ED: erectile dysfunction.

## Data Availability

The data could not be made available on open access; informed consent was obtained from all individual participants included in the study in which the open access may affect the concerns of patient privacy.

## References

[1] Zhang J., Zhang X., Cai Z., Li N., Li H. (2019). The lifetime risk and prognosis of chronic prostatitis/chronic pelvic pain syndrome in the middle-aged Chinese males. *American Journal of Men's Health*.

[2] Zhang J., Liang C., Shang X., Li H. (2020). Chronic prostatitis/chronic pelvic pain syndrome: a disease or symptom? Current perspectives on diagnosis, treatment, and prognosis. *American Journal of Men's Health*.

[3] Anderson R. U., Wise D., Sawyer T., Chan C. A. (2006). Sexual dysfunction in men with chronic prostatitis/chronic pelvic pain syndrome: improvement after trigger point release and paradoxical relaxation training. *Journal of Urology*.

[4] Johannes C. B., Araujo A. B., Feldman H. A., Derby C. A., Kleinman K. P., McKinlay J. B. (2000). Incidence of erectile dysfunction in men 40 to 69 years old: longitudinal results from the Massachusetts male aging study. *Journal of Urology*.

[5] Dutkiewicz S., Skawinski D., Duda W., Duda M. (2012). Assessing the influence of benign prostatic hyperplasia (BPH) on erectile dysfunction (ED) among patients in Poland. *Central European Journal of Urology*.

[6] Braun M. H., Sommer F., Haupt G., Mathers M. J., Reifenrath B., Engelmann U. H. (2003). Lower urinary tract symptoms and erectile dysfunction: co-morbidity or typical "aging male" symptoms? Results of the "Cologne Male Survey". *European Urology*.

[7] Rosen R. C., Fisher W. A., Eardley I. (2004). The multinational Men's Attitudes to Life Events and Sexuality (MALES) study: I. Prevalence of erectile dysfunction and related health concerns in the general population. *Current Medical Research and Opinion*.

[8] Selvin E., Burnett A. L., Platz E. A. (2007). Prevalence and risk factors for erectile dysfunction in the US. *The American Journal of Medicine*.

[9] Imai A., Yamamoto H., Hatakeyama S. (2010). Risk factors for erectile dysfunction in healthy Japanese men. *International Journal of Andrology*.

[10] Hiramatsu I., Tsujimura A., Soejima M. (2019). Tadalafil is sufficiently effective for severe chronic prostatitis/chronic pelvic pain syndrome in patients with benign prostatic hyperplasia. *International Journal of Urology*.

[11] Liang C. Z., Zhang X. J., Hao Z. Y., Shi H. Q., Wang K. X. (2004). Prevalence of sexual dysfunction in Chinese men with chronic prostatitis. *BJU International*.

[12] Hao Z. Y., Li H. J., Wang Z. P. (2011). The prevalence of erectile dysfunction and its relation to chronic prostatitis in Chinese men. *Journal of Andrology*.

[13] Sonmez N. C., Kiremit M. C., Guney S., Arisan S., Akca O., Dalkilic A. (2011). Sexual dysfunction in type III chronic prostatitis (CP) and chronic pelvic pain syndrome (CPPS) observed in Turkish patients. *International Urology and Nephrology*.

[14] Gonen M., Kalkan M., Cenker A., Ozkardes H. (2005). Prevalence of premature ejaculation in Turkish men with chronic pelvic pain syndrome. *Journal of Andrology*.

[15] Elbendary M. A., El-Gamal O. M., Salem K. A. (2009). Analysis of risk factors for organic erectile dysfunction in Egyptian patients under the age of 40 years. *Journal of Andrology*.

[16] Rosen R. C., Cappelleri J. C., Smith M. D., Lipsky J., Pena B. M. (1999). Development and evaluation of an abridged, 5-item version of the International Index of Erectile Function (IIEF-5) as a diagnostic tool for erectile dysfunction. *International Journal of Impotence Research*.

[17] Li H. J., Kang D. Y. (2016). Prevalence of sexual dysfunction in men with chronic prostatitis/chronic pelvic pain syndrome: a meta-analysis. *World Journal of Urology*.

[18] Chen X., Zhou Z., Qiu X., Wang B., Dai J. (2015). The effect of chronic prostatitis/chronic pelvic pain syndrome (CP/CPPS) on erectile function: a systematic review and meta-analysis. *PLoS One*.

[19] Muller A., Mulhall J. P. (2005). Sexual dysfunction in the patient with prostatitis. *Current Opinion in Urology*.

[20] Shoskes D. A., Prots D., Karns J., Horhn J., Shoskes A. C. (2011). Greater endothelial dysfunction and arterial stiffness in men with chronic prostatitis/chronic pelvic pain syndrome—a possible link to cardiovascular disease. *Journal of Urology*.

[21] Adams M., Sabate J. (2019). Sexual dimorphism in cardiovascular disease risk and risk factors among vegetarians: an exploration of the potential mechanisms. *Current Atherosclerosis Reports*.

[22] Berghuis J. P., Heiman J. R., Rothman I., Berger R. E. (1996). Psychological and physical factors involved in chronic idiopathic prostatitis. *Journal of Psychosomatic Research*.

[23] Oksuz E., Malhan S. (2005). The prevalence of male sexual dysfunction and potential risk factors in Turkish men: a web-based survey. *International Journal of Impotence Research*.

[24] Sprague A. H., Khalil R. A. (2009). Inflammatory cytokines in vascular dysfunction and vascular disease. *Biochemical Pharmacology*.

[25] Tran C. N., Shoskes D. A. (2013). Sexual dysfunction in chronic prostatitis/chronic pelvic pain syndrome. *World Journal of Urology*.

[26] Mo M. Q., Long L. L., Xie W. L. (2014). Sexual dysfunctions and psychological disorders associated with type IIIa chronic prostatitis: a clinical survey in China. *International Urology and Nephrology*.

[27] Riegel B., Bruenahl C. A., Ahyai S., Bingel U., Fisch M., Lowe B. (2014). Assessing psychological factors, social aspects and psychiatric co-morbidity associated with chronic prostatitis/chronic pelvic pain syndrome (CP/CPPS) in men -- a systematic review. *Journal of Psychosomatic Research*.

[28] Atlantis E., Sullivan T. (2012). Bidirectional association between depression and sexual dysfunction: a systematic review and meta-analysis. *The Journal of Sexual Medicine*.

[29] Mehik A., Hellstrom P., Sarpola A., Lukkarinen O., Jarvelin M. R. (2001). Fears, sexual disturbances and personality features in men with prostatitis: a population-based cross-sectional study in Finland. *BJU International*.

[30] Bonierbale M., Lancon C., Tignol J. (2003). The ELIXIR study: evaluation of sexual dysfunction in 4557 depressed patients in France. *Current Medical Research and Opinion*.

[31] Aubin S., Berger R. E., Heiman J. R., Ciol M. A. (2008). Original research—sexual pain disorders: the association between sexual function, pain, and psychological adaptation of men diagnosed with chronic pelvic pain syndrome type III. *The Journal of Sexual Medicine*.

[32] Cho B. L., Kim Y. S., Choi Y. S. (2003). Prevalence and risk factors for erectile dysfunction in primary care: results of a Korean study. *International Journal of Impotence Research*.

[33] Zhang X., Yang B., Li N., Li H. (2017). Prevalence and risk factors for erectile dysfunction in Chinese adult males. *The Journal of Sexual Medicine*.

